# Effective of Smart Mathematical Model by Machine Learning Classifier on Big Data in Healthcare Fast Response

**DOI:** 10.1155/2022/6927170

**Published:** 2022-02-23

**Authors:** Mahmoud Ahmad Al-Khasawneh, Amal Bukhari, Ahmad M. Khasawneh

**Affiliations:** ^1^School of Information Technology, Skyline University College, University City Sharjah, 1797 Sharjah, UAE; ^2^College of Computer Science and Engineering, University of Jeddah, Saudi Arabia; ^3^Department of Cybersecurity, Amman Arab University, Amman 11953, Jordan

## Abstract

In the past few years, big data related to healthcare has become more important, due to the abundance of data, the increasing cost of healthcare, and the privacy of healthcare. Create, analyze, and process large and complex data that cannot be processed by traditional methods. The proposed method is based on classifying data into several classes using the data weight derived from the features extracted from the big data. Three important criteria were used to evaluate the study as well as to benchmark the current study with previous studies using a standard dataset.

## 1. Introduction

One of the important areas in artificial intelligence is machine learning. The discovery of the race is the main goal of machine learning, in addition to making smart decisions. There are a lot of algorithms for machine learning, and they are mainly classified into two types and supervised, and the second category is unsupervised, and there is a class between them called semisupervised [1]. When there is big data, machine learning will be expanded by algorithms. Some researchers classify machine learning according to the categorized outputs such as regression, clustering, and density estimation, which mostly depend on teaching the decision tree, teaching the rules of association and artificial neural networks [2, 3].

Supervised algorithms include Naïve Bayes, boost algorithm, and support vector machines (SVM) that can be learned. Unsupervised learning takes undefined data and categorizes it based on features extracted and compared between them [4].

Big data is used in machine learning, which is a huge volume of structured or unstructured data. In which traditional methods are unable to process or by using traditional database methods, big data plays an active role in scientific discoveries that depend on creating values, as well as massive parallel processing, distributed file systems, cloud computing, and the use of big data technologies such as Hadoop and server database SQL [5].

Big data originally shows the size, speed, and types of data, in addition to the time of production of that data by health care providers, and includes information related to patient care, and the magnitude comes from the abundance of its production and analysis. Demographics play the role of big data, diagnoses, medical treatments, drugs, lab results, and X-ray images. In the development taking place in the electronic renaissance, sensors, and flow tools, health care data has become of interest, despite the large amount of data it contains. Healthcare data is very useful in drug discovery, medical applications, disease prediction, and so on. Big health data plays an effective role in health care, scientific research, social networks, industry, and public administration. As for big data, it is mainly categorized in the form of 5Vs as follows [6, 7]:

- Volume: large volume refers to big data. Big data contains a huge amount of information such as high-resolution videos, images, and text, in a healthcare database; the data must be processed with traditional enhanced techniques for processing images, personal information, and readings from biometric sensors, which increases the complexity of the data due to the cumulative processing.
- Velocity: velocity represents the rate of creation of large stored data. The growth rate of paper data in social networking sites and public health is increasing, and because of the diversity as well, the processing speed should be concerned with X-ray films and text data.
- Variety: big data includes a variety of data that undoubtedly requires a special type of processing, such as formatted data, Excel, or CSV data that is stored in text files, such as doctor's prescriptions, clinical data, and office records.
- Veracity: it is the validity of the data that has no real errors, which is the ability to understand health care data and its quality in addition to verifying the testimony of information such as treatment, prescription, results, and procedures.
- Value: big data takes into account the actual value of the generated data. Cost changes the importance of the value of data. Therefore, in health care, data and its cost are an actor in the system. High value to patients is the primary goal in health care.

## 2. Related Work

When thinking about machine learning, it means solving problems related to nontraditional ways. As for the data that is unusual, it is the big data that has properties that prevent it from being processed in traditional ways [8]. Big data needs a difficult and not natural prediction process, especially when we encounter abnormal data that needs to take special measures. The production of big data needs continuity of processing due to a small change in the data series that gives wrong results in the near future [9]. Academics are keen to keep track of big data and the technologies that deal with it, especially artificial intelligence. Machine learning includes working methods such as decision tree, SVM, Naïve classifier, industrial networking, clustering, and genetic computing [10, 11], all with one goal, which is to get future decisions and predictions, and with the goal of smart decisions for a machine learning strategy [12].

Big data analysis and processing are very important at the present time due to the development in information technology and the Internet. It provides in an equal way the use of computational and measurable data by machine learning of structured and unstructured data [13]. The problems with big data are not many if innovation and skill are combined. Big data may be in the biometric indicators in the google scholar through information such as the author's name, university, nationality, language, and number of references, and through the analyses of the above information, complex maps of the progress of the indexed process can be created [14]. In the world of data, there is an increase in the rate of production nowadays, so the term big data was introduced. Therefore, analyzing such data has become one of the necessities that scientists have been finding compatible algorithms with [15]. Here, we will take a historical overview about big data and its relationship with machine learning and algorithms that were presented in previous studies as in Figure 1.

Big data analytics are associated with the work of large organizations and the areas of innovation and competitive production. We can define them as techniques deployed to reveal the hidden patterns of understanding the work contexts through the output. Each researcher divides machine learning according to how it works and how closely the topic relates to the main idea. Classification in this research focuses on machine learning and its classifications related to big data. Basically, classifications consist of many algorithms, but the most important of them are CVM, KNN, and ELM [16]. All are considered features extracted from the data in advance to be indexed based on certain criteria in the algorithm. The second and important category is the aggregation, which consists of several algorithms, but the main ones that work with big data are the *K*-Mean and DPSCAN algorithm [17], which depends on the relationship of the data with each other and the extent of the impact of one on the other. As for the last type, the Volitional Algorithm, it is widely used with data that has an interactive nature, meaning that the big data is continuously updated over time. Such algorithms are not useful in the medical field, which deals with data of great importance to human lives, especially those that rely on unanimous decisions due to the seriousness of the situation. Among these algorithms are GA, ACO, and PSO [18]. As conclusion many algorithms suggested in literature, each has advantage and disadvantage so that we try to adapt algorithm with minimum errors.

## 3. Big Data and Machine Learning

Big data applications are important in our daily lives. Among these applications is health care for patients that need to manage their data, especially with the spread of epidemics at the present time.

### 3.1. Big Data in Healthcare

According to IDC reports, the growth of big data in healthcare is expected to accelerate compared to other areas such as industries, financial services, and media. Health care data is expected to reach 36% until 2025, according to projections Compound Annual Growth Rate (CAGR) [19]. The global big data market is expected to reach $34.27 billion in healthcare in 2022 if the current annual growth rate continues at 22%, which will reach the health sector with a budget of $68 billion [20], so focusing on this area will save billions of dollars which is the main objective in this research. Big data in health care take the data from different resources as shown in Figure 2

Some resources provide data online that some time increased exponentially by the time, and most of the data comes from the document of hospital or patient himself. Big data in the field of health care comes from several sources, starting from electronic records, search engines, and sensors, thus obtaining endless data that needs processing and analysis to know its use in the correct way. From this point of view, the usefulness of medical big data is at all levels, from the patient to the hospital and to society in general.

### 3.2. Machine Learning

Machine learning is considered a part or branch of artificial intelligence, which refers to the ability of information technology systems to find the best solutions for multiple patterns in big data. Machine learning depends on deducing algorithms and solutions in several courses and choosing the best among them. Machine learning algorithms rely on prior data extracted from master data called features [21]. Synthetic knowledge is derived from experiences in machine learning. For machine learning, statistical methods and mathematical processes are used in order to exploit computer resources as a whole.

Specifically, the computer program learns from experience (*E*) while executing some tasks (*T*) in order to measure performance (*P*), all of this to improve performance and get better results. The summary of the work is that the computer program can learn to improve performance, and therefore, it can be measured for some tasks through experience. The number of resources within big data needs some processes to get performance *p*_+1_ which is smaller than *P*_*i*_ such as {*P*_*i*_, *P*_*i*+1_} ⊂ *P* to get experience of *E* in the context of {*e*_*i*_, *e*_*i*+1_} ⊂ *E*, respectively. Then, the machine learning model is aimed at improving each performance till exceeding all iterations in the tasks. ML has basically four paradigms as shown in Figure 3 with brief summarization.

- Unsupervised model is an experiment that contains many features of big data in order to identify the useful properties of group structuring, and in the field of machine learning, knowing the distribution possibilities is of great importance in order to choose the right group with high impact, and clustering is an example of unsupervised learning models [22]
- Supervised model is the experience of a set of data that contains features, but these features are related to a specific label or goal. The label is either binary (0 and 1) and indexed on the basis of their proximity to the correct output, or they are pretrained, and thus, new data is checked based on prior training [23]
- Semisupervised model is a homogeneous mixture of supervised and unsupervised models to obtain an individual accurate result for the specific tasks. Sometimes, it is called transformative education or inductive education [24]
- Reinforcement depends on interaction with the environment and the work itself by feeding back learning and acquiring new real-time experiences [25]

On the basis of these models, the linkage is revealed in the privacy of each of them. In general, the supervised and unsupervised models are trained on tasks (*T*) in the data that produce temporary jobs during implementation. Improving performance (*P*) is the main goal in some tasks. Training on real-time data that comes directly from the user is somewhat sensitive as in social media and contains privacy. Therefore, machine learning detects future privacy intentions, which is the goal of this study.

### 3.3. Challenging of Machine Learning in Big Data

There are many challenges related to the use of machine learning techniques in big data, including the following: (1) flexibility of computational design and the ability to develop machine learning through it; (2) through machine learning algorithms, being able to understand the characteristics and importance of data before applying the algorithm; and (3) ability to learn and build architecture and adapt to increasing volumes of labeled data.

Among the problems that we face when using machine learning with big data, which sometimes makes it inappropriate [26], are as follows: (1) The first one is not adapting to the data, which means that some algorithms are suitable for certain data and not suitable for other data. (2) Training, which depends on a machine learning algorithm, uses dataset labeled for classification, and dataset that does not have label is inaccurately classified. (3) A particular algorithm may be good for certain data and bad for other data. One of the most important challenges facing machine learning is to expand the scope of big data to appropriate dimensions [8, 27, 28]. There are challenges related to the speed of data processing, as machine learning algorithms need time to train before starting the actual processing. Therefore, machine learning algorithms are designed based on the ability to analyze and the type of data to be processed.

To increase the efficiency of the system's work, the data is redesigned using SMART PLS that first classifies the data before starting to implement the machine learning algorithm.

## 4. Materials and Methods

Machine learning depends on its work on two methods; the first and the most important method is the classification process. Big data is initially initialized and indexed into aggregates and by master key. Big data analysis is preliminary, such as *s*(*bigdata* *analytic*) < min(*s*(*bigdata*), *s*(*analytic*) = *s*(*v*_1_⋁ *v*_2_), where *s* is a group of data, ⋁ is *or* operation, and *v* is considered the value sequence. Let *v*_1_, *v*_2_, *v*_3_ ∈ *V* where *V* is the big data value; then *s*(*v*_1_) = *F*(*v*_1_), *s*(*v*_2_) = *F*(*v*_2_) and *s*(*v*_3_) = *F*(*v*_3_), so the main function will be like

(1) $$\begin{array}{c} s\left(v_{1}\vee v_{2}\right)=s\left(v_{1}\right)\cap s\left(v_{2}\right)=F\left(v_{1}\right)\cap F\left(v_{2}\right). \end{array}$$

By Equation (1), we can cluster the big data into subgroups with its function and using SMART PLS program to calculate the weights that can help at the next step of analytics. Statistical program was used to arrange the data into appropriate sections for better preparation. Due to *s*(*v*_*i*_), *i* = {1, 2, 3, ⋯, *n*, ⋯}, then the whole group of big data is illustrated in

(2) $$\begin{array}{c} s\left(v_{1}⋁v_{2}⋁v_{3}\cdots ⋁v_{n}\right)=\overset{n}{\underset{1}{\prod }}F\left(v_{i}\right)=F\left(v_{1}\right)\cap F\left(v_{2}\right)\cap \cdots F\left(v_{n}\right). \end{array}$$

This make relation of the entire big data within a subgroup achieve *n* groups clustered in certain condition. And because of data availability that will be still updated or online produced, the limit of *n* will change to infinity

(3) $$\begin{array}{c} s\left(v_{1}⋁v_{2}⋁v_{3}\cdots ⋁v_{n}\cdots \right)=\overset{\infty }{\underset{1}{\prod }}F\left(v_{i}\right). \end{array}$$

And with respect to the operation *or* (∨) in case of updated data, but when produced, new data belong to original big data operation *or* will change to *and* (∧) as

(4) $$\begin{array}{c} s\left(v_{1}\wedge v_{2}\wedge v_{3}\cdots \wedge v_{n}\right)=\overset{n}{\underset{1}{\prod }}F\left(v_{i}\right)=F\left(v_{1}\right)\cup F\left(v_{2}\right)\cup \cdots F\left(v_{n}\right), \end{array}$$

(5) $$\begin{array}{c} s\left(v_{1}\wedge v_{2}\wedge v_{3}\cdots \wedge v_{n}\cdots \right)=\overset{\infty }{\underset{1}{\prod }}F\left(v_{i}\right). \end{array}$$

This process occurs in preparation data or initialization stage after the big data will be ready to extract features as shown in Figure 4.

Patient behavior was predicted by using linear predictor for *j* data point such as *j* = 1, 2, 3, .., *n*.

(6) $$\begin{array}{c} f\left(j\right)=a_{0}+a_{1}x_{j1}+a_{2}x_{j2}+\cdots +a_{m}{\text{x}}_{jm}. \end{array}$$

In the above equation, *x*_*j*_ is the feature vector for *j* = 1, 2, ⋯, *m* of *m*-th interactive variable of data point value *j*, and *a*_0_, *a*_1_, *a*_2_, ⋯, *a*_*m*_ are the coefficients of the results that presentative relation between the data since the coefficient is accumulative into the vector. Feature extraction based on *j*-th cluster of *M* features *<x*_1_, *x*_2_, ⋯, *x*_*n*_ *>* such as n refer to cluster number. Weight that controls the features *<w*_1_, *w*_2_, ⋯, *w*_*m*_ *>* was also used to calculate $\bar{x}$ of mean value belonging to feature *x*

(7) $$\begin{array}{c} \bar{x}=\frac{1}{N}\overset{N}{\underset{i=1}{\sum }}x_{i}. \end{array}$$

From above equation, we can get the standard deviation *σ* shown in

(8) $$\begin{array}{c} \sigma =\sqrt{\frac{\sum_{i=1}^{N}\left(x_{i}^{j}-x^{-j}\right)}{N-1}}. \end{array}$$

Standard deviation was related to new features of certain weight and expressed as

(9) $$\begin{array}{c} {\bar{x}}_{i}=\frac{x_{i}}{\sigma }. \end{array}$$

Then, weight can be calculated as

(10) $$\begin{array}{c} w_{i}=\frac{1}{\sigma }. \end{array}$$

Figure 5 shows behavior of classifier when weight value is variable including some conditions.

Big data will train (*x*_*i*_, *y*_*i*_) for *N* iteration to *i*, with *x*_*i*_ ∈ *R* and *y*_*i*_ ∈ {−1, 1}, of learning classifier *Y* such that

(11) $$\begin{array}{c} Y=\left\{\begin{array}{c} +1,\;\text{if }x_{i}\in \text{class }A,\\ -1,\;\text{if }x_{i}\in \text{class }B. \end{array}\right. \end{array}$$

The classification of the data is in a sequential form, and this sequence can be rearranged in the event that there are cutoffs, such as updating the data or adding supplementary data to the previous data. In Results and Discussion, we will discuss training and data testing and the method of implementing the classifier for big data.

## 5. Results and Discussion

The proposed algorithm was implemented using MATLAB language and Windows 10 operating system on standard dataset called UCI ML [29] and with a 50 of attributes as in Table 1

The dataset consisted of 50 attributes with 101,767 patient records. The processing was calculated and divided into two parts: the first section is training, with 80%, with the data that contains a label, and the second section is testing, with 20%. The first big dataset reduced into 20123 records when applying reduce procedure to be the best fit dataset even though some attributes also reduced for parallel execution [30, 31], after reducing some attributes in dataset highlighted such as gender, age, medical specialty, time in hospital, and weight, as shown in Figure 6.

We check the validity and reliability of the database attributes within the algorithms to find the relation among the data during processing to take effect of certain attributes. Such as {*weight*, *age*}⟶{*num* *emergency*}. Classification process is done by multiclass technique to find three main evaluation factors such as precision, probability of detection, and *F*-score. And for benchmark results, then, we used standard dataset and each algorithm contains different result values, so efficiency of the proposed method is illustrated in the Table 2.

Better classification rate achieved due to reducing data was great, and the features extracted were useful, so predictions are classified as two cases correctly and incorrectly; many conditions were applied during creating confusion matrix such as probability of detection (sensitivity), accuracy, precision, true negative rate (specificity), and *F*-score [32]. The true positive detection occurs during emergency classification; then accuracy is formulated as ratio in confusion matrix. Equations below refers to criteria that can be detected by the proposed algorithm.

(12) $$\begin{array}{c} \text{Accuracy}=\frac{\left(\text{TP}+\text{TN}\right)}{\left(\text{TP}+\text{FP}+\text{FN}+\text{TN}\right)},\\ \text{Probability of detection}=\frac{\text{TP}}{\left(\text{TP}+\text{FN}\right)},\\ \text{True Negative}=\frac{\text{TN}}{\text{FP}+\text{TN}},\\ \text{Precision}=\frac{\text{TP}}{\text{TP}+\text{FP}}, \end{array}$$

where TP represents the count of emergency case classified as emergent patient, TN refers to normal classified, FP refers to the number of emergent case, and FN refers to the number of normal classified. Most of results depend on confusion matrix and its condition as shown in Table 3.

In Table 3, TP refers to True Position, TN refers to True Negative, FP refers to False Position, and FN refers to False Negative. In addition, these criterion measurement classifiers can also be doing additional aspects such as robustness, speed, scalability, and interpretability.

## 6. Conclusion

The evaluation of big data is often useful for health care, which has received high interest nowadays due to the spread of viruses and epidemics in general. The data coming from the field of health care in general is of two types, either updateable or in the form of large data. Classifying such data requires a complex computational process and the development of a classifier adaptable to that data. In this study, a classifier was improved based on the weight of the data, and this weight is derived from the extracted features in order to classify the medical data and according to the importance. At first, the data is reduced in order to be processed as quickly as possible, and then it is classified on the basis of several types. The main attributes such as age, medical prescription, number of visits to the doctor, hospitalization periods, medical analyses, and others are considered complementary relationships for classification. The study was evaluated by three criteria: precision, probability of detection, and *F*-score used for benchmarking on standard dataset; meanwhile, other evaluations such as accuracy and true negative are also considered in this study.

## Figures and Tables

**Figure 1:** Structure of big data related to machine learning in existing studies.

**Figure 2:** Big data health care resources.

**Figure 3:** Type of ML paradigms.

**Figure 4:** Big data process within ML.

**Figure 5:** Classification underweight condition.

**Figure 6:** Database attributes after reducing.

**Table 1:** Attribute within UCI ML dataset.

encounter_id	patient_nbr	Race
Gender	age	Weight
admission type id	discharge disposition id	admission_source_id
time_in_hospital	payer_code	medical_specialty
numb_lab_procedures	num_procedures	num_medications
number_outpatient	number_emergency	number_inpatient
diag_1	diag 2	diag 3
number_diagnoses	max_glu_serum	AlCresult
Metformin	repaglinide	Nateglinide
Chlorpropamide	glimepiride	Acetohexamide
Glipizide	glyburide	Tolbutamide
Pioglitazone	rosiglitazone	Acarbose
Migitol	troglitazone	Tolazamide
Examide	citoglipton	Insulin
glyburide-metformin	glipizide-metformin	glimepiride-pioglitazone
metformin-rosiglitazone diabetesMed	metformin-pioglitazone readmitted	Change

**Table 2:** Evaluation criteria.

Parameters	Proposed weighted classification	DT outlier	DTI	RBF
Precision	0.99	0.99	0.89	0.82
Probability of detection	0.76	0.7	0.65	0.87
*F*-score	0.83	0.82	0.73	0.84

**Table 3:** Confusion matrix.

Predicted class				
Actual class		Yes	No	Total
	Yes	TP	FN	*P*
	No	FP	TN	*N*
	Total	*P*′	*N*′	*P* + *N*

## Data Availability

The data used to support the findings of this study are available from the corresponding author upon request.
